# Anti-inflammatory effects of Hwang-Heuk-San, a traditional Korean herbal formulation, on lipopolysaccharide-stimulated murine macrophages

**DOI:** 10.1186/s12906-015-0971-2

**Published:** 2015-12-23

**Authors:** Hye Joo Kang, Su Hyun Hong, Kyung-Hwa Kang, Cheol Park, Yung Hyun Choi

**Affiliations:** Department of Biochemistry, Dongeui University College of Korean Medicine, 52-57, Yangjeong-ro, Busanjin, Busan, 614-052 Republic of Korea; Anti-Aging Research Center, Dongeui University, 176 Eomgwangno Busanjin-gu, Busan, 614-714 Republic of Korea; Department of physiology, College of Korean Medicine, Dongeui University, Busan, 614-714 Republic of Korea; Department of Molecular Biology, College of Natural Sciences, Dongeui University, 176 Eomgwangno Busanjin-gu, Busan, 614-714 Republic of Korea

**Keywords:** Hwang-Heuk-San, RAW 264.7 macrophage, anti-inflammation, MAPKs, NF-κB/AP-1

## Abstract

**Background:**

Hwang-Heuk-San (HHS), a Korean traditional herbal formula comprising four medicinal herbs, has been used to treat patients with inflammation syndromes and digestive tract cancer for hundreds of years; however, its anti-inflammatory potential is poorly understood. The aim of the present study was to investigate the anti-inflammatory effects of HHS using a lipopolysaccharide (LPS)-activated RAW 264.7 macrophage model.

**Methods:**

The inhibitory effects of HHS on LPS-induced nitric oxide (NO), interleukin-1β (IL-1β) and tumor necrosis factor-α (TNF-α) production were examined using Griess reagent and enzyme-linked immunosorbent assay (ELISA) detection kits. The effects of HHS on the expression of inducible NO synthase (iNOS), IL-1β and TNF-α, their upstream signal proteins, including nuclear factor κB (NF-κB), mitogen-activated protein kinases (MAPKs), and activator protein (AP-1), were also investigated.

**Results:**

A noncytotoxic concentration of HHS significantly reduced the production of NO, IL-1β and TNF-α in LPS-stimulated RAW 264.7 cells, which was correlated with reduced expression of iNOS, IL-1β and TNF-α at the mRNA and protein levels. HHS efficiently blocked the phosphorylation of MAPKs, especially that of extracellular signal-regulated kinase (ERK) and c-Jun NH2-terminal kinase (JNK) but not that of the p38 MAPK. The reduced production of inflammatory molecules by HHS was followed by decreased activity of NF-κB and AP-1.

**Conclusions:**

These results suggest that HHS may offer therapeutic potential for treating inflammatory diseases accompanied by macrophage activation.

## Background

There is increasing awareness that inflammation is a natural defense system found in the human body and that it plays a major role in the pathogenesis of many inflammatory disorders [1, 2]. Although macrophages are important in the host-defense mechanism, pathogen-induced overproduction of inflammatory factors from macrophages and cellular damage-derived inflammation-inducing molecules have been implicated in inflammation-related diseases, such as arthritis, inflammatory bowel diseases, and asthma [3].

Accumulating evidence indicates that specific stimuli, such as the endotoxin lipopolysaccharide (LPS), a component of the outer membrane of gram-negative bacteria, give rise to the activation of macrophages and result in the secretion of a number of different proinflammatory mediators and cytokines, including nitric oxide (NO), interleukin-1β (IL-1β) and tumor necrosis factor-α (TNF-α) [3–5]. LPS can bind to toll-like receptor 4 (TLR4), which is expressed on macrophages. This complex activates various cellular signaling events, including mitogen-activated protein kinases (MAPKs), and subsequently induces the activation of various transcription factors, such as nuclear factor (NF)-κB and activator protein (AP-1) [6, 7].

MAPKs, extracellular signal regulated kinase (ERK), c-Jin NH2-terminal kinase (JNK), and p38 MAPK are a group of signaling molecules that also play an important role in relaying inflammatory information from the extracellular space to the cytoplasm and nucleus to modulate inflammatory responses [7, 8]. Phosphorylation-induced activation of MAPKs is known to be a critical component in the production of proinflammatory molecules in activated macrophages. Previous studies have shown that TLR4-induced activation of MAPKs resulted in the activation of the nuclear translocation of NF-κB and AP-1 and, finally, the initiation of proinflammatory responses [9, 10]. Under normal physiological conditions, NF-κB dimmers of p50 and p65 subunits are present in the cytoplasm and attached to the suppressor protein inhibitor of NF-κB (IκB). NF-κB activation occurs *via* phosphorylation and subsequent activation of MAPKs, followed by degradation of IκB bound to NF-κB, resulting in the translocation of NF-κB from the cytoplasm to the nucleus to promote the expression of various proinflammatory genes [6, 11]. AP-1 is an important regulator of gene expression involved in inflammation activation, and it forms heterodimer complexes with c-Jun and c-Fos. Various factors, including growth factors, cytokines, and stress, induce AP-1 [7, 8]. AP-1 is activated by TLR agonists and cytokines, dependent on the activation of MAPKs. Therefore, treatments aimed at inhibiting MAPKs and NF-κB, as well as AP-1, may have potential therapeutic advantages as anti-inflammatory agents [12, 13].

For thousands of years, herbal medicines have been used with apparent safety and efficacy for alleviating and treating various diseases in many countries. Recently, there has been increasing interest in the pharmacological activity of traditional herbal formulas that are widely used in traditional medicine in East Asia, including Korea, China, and Japan, and numerous studies support their potential clinical benefit for diseases that are difficult to treat [14, 15]. Typical traditional Korean medicinal prescriptions derived from ancient Chinese herbal medicines consist of more than four components that are mixed to minimize side effects, maximize medical effects, and improve the patient’s quality of life [16, 17]. Among them, Hwang-Heuk-San (HHS) is an aqueous polyherbal formulation comprising four medicinal herbs (Table 1). HHS has been used to treat patients with inflammation syndromes and digestive tract cancer in traditional Korean medicine. Despite its valuable clinical effects on patients, little is known about the molecular pharmacological basis of the effects of HHS. In this study, as part of our ongoing screening program to evaluate the anti-inflammatory potential of new compounds from traditional medicinal resources, we investigated the impact of HHS on the inflammatory response of LPS-challenged RAW 264.7 macrophages, as well as the signaling pathways involved in these processes. Our data suggest that HHS inhibits LPS-induced NO, IL-1β and TNF-α production in RAW 264.7 cells, at least in part, through blockade of the NF-κB, MAPK, and AP-1 signaling pathways.

**Table 1:** Herbal components and amount of HHS decoction

Herbal medicine (pharmacognostic nomenclature)	Raw material amount (g/%)
*Rheum palmatum* L. (Rhei Radix et Rhizoma)	36.0 (47.4)
*Psoralea corylifolia* L. (Psoraleae Fructus)	16.0 (21.0)
*Pharbitis nil* Chois. (Pharbitidis Semen)	16.0 (21.0)
*Arctium lappa* L. (Arctii Fructus)	8.0 (10.5)
Total amounts	76 (100)

## Methods

### Materials and reagents

Dulbecco’s modified Eagle's medium (DMEM) and fetal bovine serum (FBS) were purchased from WelGENE Inc. (Daegu, Republic of Korea). LPS (*Escherichia coli* Serotype 055:B5), 3-[4,5-dimethylthiazol-2-yl]-2,5-diphenyltetrazolium bromide (MTT), and Griess reagent were from Sigma-Aldrich Chemical Co. (St. Louis, MO, USA). Mouse IL-1β and TNF-α enzyme-linked immunosorbent assay (ELISA) detection kits, and enhanced chemiluminescence (ECL) detection system were purchased from R&D Systems (Minneapolis, MN, USA) and Amersham Co. (Arlington Heights, IL, USA), respectively. Various primary and secondary antibodies for Western blot analysis were purchased from Cell Signaling Technology, Inc. (Boston, MA, USA) and Santa Cruz Biotechnology (Santa Cruz, CA, USA). All other chemicals were purchased from Sigma-Aldrich Chemical Co.

### Preparation of the HHS

The four medicinal herbs forming HHS were obtained from Dongeui Oriental Hospital, Dongeui University College of Korean Medicine (Busan, Republic of Korea). The origin of the medicinal herbs was confirmed taxonomically by Professor Su Hyun Hong, Dongeui University College of Korean Medicine (Busan, Republic of Korea). Each of the four herbs in HHS was cut into small pieces and then mixed together to obtain a total amount of 76 g in the ratios shown in Table 1. The mixture was boiled with distilled water (76 g/500 ml) for 3 h. The extract solution was filtered using a 0.45-mM filter to remove insoluble materials, and the blended supernatants were lyophilized and then crushed into a thin powder (yield = 21 % w/w, dried extract/crude herb). The dried extract was dissolved to a 100 mg/ml concentration with distilled water before use, and the stock solution was then diluted with medium to the desired concentration prior to use.

### Cell culture and LPS stimulation

A murine macrophage cell line RAW 264.7 was obtained from the American Type Culture Collection (Manassas, VA, USA) and grown in DMEM containing 10 % FBS, 100 U/ml of penicillin, and 100 mg/ml of streptomycin in an incubator at 37 °C, 5 % CO_2_, and 95 % humidity. To stimulate the cells, the medium was exchanged with fresh DMEM, and LPS (100 ng/ml) was added in the presence or absence of HHS for the indicated periods.

### Assessment of cell viability

The effects of HHS on cell viability were evaluated using a colorimetric MTT assay. In brief, the RAW 264.7 cells were seeded at a density of 1 × 10^4^ cells/well in a 96 well-plate, incubated at 37 °C for 24 h, and treated with various concentrations of HHS alone or with LPS (100 ng/ml). After incubation for 24 h, the medium was discarded, and MTT solution was added to each well and incubated for another 3 h at 37 °C. The medium was discarded, and dimethyl sulfoxide was added to dissolve the formazan dye. The optical density was the read at 450 nm using an ELISA reader (Infinite M200, Tecan, Männedorf, Switzerland).

### Measurement of NO production

The accumulation of NO was assayed using Griess reagent. In brief, the cells were pretreated with different concentrations of HHS for 1 h and stimulated with LPS for 24 h. Then, 100 μl of the Griess reagent were mixed with an equal volume of cell supernatant and incubated at room temperature for 5 min. The optical density at 540 nm was measured, and the concentration of nitrite was calculated according to the standard curve generated from known concentrations of sodium nitrite [18].

### IL-1β and TNF-α immunoassay

After treatment with HHS in the presence or absence of LPS, the levels of IL-1β and TNF-α in the culture media were quantified using ELISA kits according to the manufacturer’s instructions. The absorbance was read at a wavelength of 450 nm using a microplate reader [19].

### RNA isolation and reverse transcriptase polymerase chain reaction (RTPCR)

Total RNA was isolated using TRIzol reagent (Invitrogen Life Technologies, Carlsbad, CA, USA) according to the manufacturer’s instructions and reverse transcribed using MMLV reverse transcriptase (Promega, Madison, WI, USA) to produce cDNAs. RT-generated cDNAs encoding *iNOS, IL-1β* and *TNF-α* genes were amplified by PCR using selective primers (Table 2), which were purchased from Bioneer (Seoul, Republic of Korea). Thermal cycling was carried out for 30 s at 95 °C, followed by 40 cycles of 5 s at 95 °C, and 30 s at 60 °C. Following amplification, the PCR reactants were electrophoresed in 1 % agarose gels and visualized by ethidium bromide (EtBr) staining. In a parallel experiment, glyceraldehyde-3-phosphate dehydrogenase (GAPDH) was used as an internal control [20].

**Table 2:** Primers of targeted genes

Targeted genes		Primer sequences
iNOS	Sence Antisence	5'-ATGTCCGAAGCAAACATCAC-3' 5'-TAATGTCCAGGAAGTAGGTG-3
IL-1β	Sence Antisence	5'-ATGGCAACTGTTCCTGAACTCAACT-3' 5'-TTTCCTTTCTTAGATATGGACAGGAC-3'
TNF-α	Sence Antisence	5'-CATCTTCTCAAAATTCGAGTGACAA-3' 5'-TGGGAGTAGACAAG GTACAACCC-3'
GADPH	Sence Antisence	5'-TGGCAAAGTG GAGATTGTTGC-3' 5'-AAGATGGTGATGGGCTTCCCG-3'

### Western blot analysis

The cells were washed and scraped into cold phosphate-buffered saline (PBS) and centrifuged at 500 × g at 4 °C. The cell pellets were resuspended in lysis buffer (20 mM sucrose, 1 mM ethylenediaminetetraacetic acid, 20 μM Tris-HCl, pH 7.2, 1 mM dithiothreitol, 10 mM KCl, 1.5 mM MgCl_2_, and 5 μg/ml aprotinin). After cell debris was discarded following centrifugation at 13,000 g for 15 min, the protein concentration was determined using a Bio-Rad kit (Bio-Rad Laboratories, Hercules, CA, USA). In a parallel experiment, nuclear and cytosolic proteins were prepared using nuclear extraction reagents (Pierce Biotechnology, Rockford, IL, USA) according to the manufacturer’s protocol. Equal amounts of protein from each sample were separated by sodium dodecyl sulfate (SDS)-polyacrylamide gel electrophoresis and transferred onto nitrocellulose membranes (Schleicher & Schuell, Keene, NH, USA). Nonspecific sites were blocked by the incubating membranes for 1 h at room temperature in 5 % (w/v) nonfat milk powder in Tris-buffered saline containing 0.05 % (v/v) Tween-20 (TBS-T). Thereafter, the membranes were incubated overnight at 4 °C with the corresponding primary antibodies and subsequently incubated with the appropriate secondary antibodies conjugated to horseradish peroxidase. The specific proteins were detected using an ECL detection system.

### Immunofluorescent staining for NF-κB p65

RAW 264.7 cells were seeded on glass coverslips in 6-well plates for 24 h, and the cells were treated with HHS for 1 h and then stimulated with LPS for 30 min. Then, the cells were fixed with 3.7 % paraformaldehyde in PBS for 10 min at 4 °C. The cells were incubated with 0.4 % Triton X-100 for 10 min and blocked with 5 % bovine serum albumin for 1 h, followed by probing with rabbit anti-p65 NF-κB antibody overnight at 4 °C. They were then incubated with fluorescein isothiocyanate (FITC)-conjugated donkey anti-rabbit IgG (Jackson ImmunoResearch Laboratories Inc., West Grove, PA, USA) for 2 h at room temperature. After washing with PBS, nuclei were counterstained with 4,6-diamidino-2-phenyllindile (DAPI) solution (1 mg/ml) for 15 min in the dark, and fluorescence was visualized using a fluorescence microscope (Carl Zeiss, Oberkochen, Germany) [21].

### Electrophoretic mobility assay (EMSA)

DNA-protein binding assays were carried out with nuclear extract. Briefly, the preparation of nuclear extracts was conducted using NE-PER nuclear extraction reagents (Pierce, Rockford, IL, USA). Synthetic complementary NF-κB (5'-AGT TGA GGG GAC TTT CCC AGG C-3') and AP-1 (5'-CGC TTG ATG ACT CAG CCG GAA-3') binding oligonucleotides (Santa Cruz Biotechnology) were 30-biotinylated using a biotin 30-end DNA labeling kit (Pierce) according to the manufacturer’s instructions and annealed for 30 min at room temperature. The reaction mixtures were electrophoretically separated on 4 % polyacryl-amide gels in 0.5× Tris-borate buffer and transferred to nylon membranes. The transferred DNAs were cross-linked to the membranes at 120 mJ/cm^2^ and detected using horseradish peroxidase-conjugated streptavidin (LightShift™ chemiluminescent EMSA kit, Pierce) according to the manufacturer’s instructions.

### Statistical analysis

Data from at least three independent experiments were expressed as the mean ± standard deviation (SD). Statistical comparisons between different groups were performed using a one-way ANOVA, followed by Student’s *t*-tests after comparing each treated group to the negative control. Values of *p* < 0.01 were considered statistically significant.

## Results

### HHS inhibited the release of NO and expression of iNOS in LPS-stimulated RAW 264.7 cells

NO production is a widely used indicator of macrophage activation among many inflammatory mediators. iNOS expression generated in activated macrophages mediates the synthesis of NO, which is then released into the culture medium [22, 23]. In the present study, RAW 264.7 cells were challenged with LPS in the presence or absence of HHS, and the levels of NO were measured by Griess reagent. As presented in Fig. 1a, the pretreatment with HHS concentration-dependently suppressed NO secretion, with statistical significance. Next, we investigated whether the inhibitory effect of HHS on NO production was related to the modulation of iNOS enzyme levels. Figure 1b demonstrates that HHS strongly suppressed the protein expression of iNOS compared with that of the LPS only-treated group. Furthermore, HHS markedly repressed iNOS mRNA expression in the LPS-stimulated RAW 264.7 cells (Fig. 1c), suggesting that the HHS-mediated inhibition of NO production is associated with transcriptional downregulation of the iNOS gene.

**Fig. 1:** Inhibition of NO production and iNOS expression by HHS in LPS-stimulated RAW 264.7 macrophages. The cells were pretreated with various concentrations of HHS for 1 h and then incubated with LPS (100 ng/ml) for 24 h. **a** The amount of NO production in the medium was measured using the Griess reaction. Statistical significance was determined by a one-way ANOVA (*, *p* < 0.05 vs. untreated control; ^#^, *p* < 0.05 vs. LPS-treated group). **b** Total cellular proteins (30 μg) were resolved by SDS-polyacrylamide gel electrophoresis, transferred to nitrocellulose membranes, and detected with anti-iNOS antibody and an ECL detection system. **c** After LPS treatment for 6 h, total RNA was prepared for RT-PCR analysis of iNOS gene expression. The amplified PCR products were run in 1 % agarose gel and visualized by EtBr staining. Actin and GAPDH were used as internal controls for the Western blot and RT-PCR assays, respectively

### HHS inhibited the release and expression of IL-1β and TNF-α in LPS-stimulated RAW 264.7 cells

Proinflammatory cytokines, such as IL-1β and TNF-α, produced in response to inflammatory stimuli can contribute to inflammation [3, 24]. Thus, they are regarded as targets for inhibiting the inflammatory process. To confirm the effect of HHS on the production of proinflammatory cytokines, the IL-1β and TNF-α concentration in the culture medium was measured by ELISA. Consistent with the NO results, HHS also inhibited IL-1β and TNF-α production in a concentration-dependent manner (Figs. 2a and 3b). To confirm whether the inhibition of IL-1β and TNF-α production by HHS was due to decreased IL-1β and TNF-α expression, we examined the levels of IL-1β and TNF-α mRNA and protein after treating the LPS-stimulated RAW 264.7 cells with HHS. As presented in Fig. 2b, c, 3b and c, HHS suppressed both the protein and mRNA expression of IL-1β and TNF-α in a concentration-dependent manner. These results showed that HHS was able to inhibit the expression of IL-1β and TNF-α at the transcriptional level, which, in turn, reduced the production of IL-1β and TNF-α in the LPS-stimulated RAW 264.7 cells.

**Fig. 2:** Inhibition of IL-1β production and its expression by HHS in LPS-stimulated RAW 264.7 macrophages. The cells were pretreated with various concentrations of HHS for 1 h and then incubated with LPS (100 ng/ml) for 24 h. **a** The amounts of IL-1β were measured in culture media using a commercial ELISA kit. Statistical significance was determined by a one-way ANOVA (*, *p* < 0.05 vs. untreated control; ^#^, *p* < 0.05 vs. LPS-treated group). **b** Total cellular proteins (30 μg) were resolved by SDS-polyacrylamide gel electrophoresis, transferred to nitrocellulose membranes, and detected with anti-IL-1β antibody and an ECL detection system. **c** After LPS treatment for 6 h, total RNA was prepared for RT-PCR analysis of IL-1β gene expression. The amplified PCR products were run in 1 % agarose gel and visualized by EtBr staining. Actin and GAPDH were used as internal controls for the Western blot and RT-PCR assays, respectively

**Fig. 3:** Inhibition of TNF-α production and its expression by HHS in LPS-stimulated RAW 264.7 macrophages. The cells were pretreated with various concentrations of HHS for 1 h and then incubated with LPS (100 ng/ml) for 24 h. **a** The amounts of TNF-α were measured in culture media using a commercial ELISA kit. Statistical significance was determined by a one-way ANOVA (*, *p* < 0.05 vs. untreated control; ^#^, *p* < 0.05 vs. LPS-treated group). **b** Total cellular proteins (30 μg) were resolved by SDS-polyacrylamide gel electrophoresis, transferred to nitrocellulose membranes, and detected with anti-TNF-α antibody and an ECL detection system. **c** After LPS treatment for 6 h, total RNA was prepared for RT-PCR analysis of TNF-α gene expression. The amplified PCR products were run in 1 % agarose gel and visualized by EtBr staining. Actin and GAPDH were used as internal controls for the Western blot and RT-PCR assays, respectively

### HHS inhibited the activation of the NF-κB pathway in RAW 264.7 macrophages upon LPS stimulation

As NF-κB plays a pivotal role in the regulation of the expression of inflammatory mediators and cytokines, it is a good target for treating inflammatory diseases. Moreover, many anti-inflammatory compounds exert their effects by inhibiting the NF-κB signaling pathway [6, 11]. Therefore, we investigated whether HHS suppressed the degradation of IκB and the nuclear translocation of NF-κB by Western blotting analysis after pretreating the cells with the indicated concentrations of HHS for 1 h and stimulated with LPS for 30 min. The treatment with LPS alone markedly increased the nuclear levels of p65, a component of the heterodimer of NF-κB, and HHS effectively blocked the LPS-induced accumulation of NF-κB p65 in the nucleus in a concentration-dependent manner (Fig. 4a). We next examined the ability of HHS to inhibit the degradation of IκBα in the cytoplasm and found that HHS promoted the cytosolic accumulation of IκBα. The immunofluorescence images also revealed that NF-κB p65 was normally sequestered in the cytoplasm, and nuclear translocation of NF-κB p65 was not observed in the cells after treatment with HHS alone in the absence of LPS stimulation (Fig. 4b). LPS stimulation significantly induced the nuclear localization of NF-κB p65 in RAW 264.7 cells, whereas pretreating the cells with HHS abolished this effect. To confirm whether HHS affected the activation of NF-κB, the DNA-binding activity of NF-κB was investigated by an EMSA. The results revealed significantly reduced DNA-binding activity of NF-κB in the nuclear extracts obtained from the LPS-activated macrophages pretreated with HHS (Fig. 4c). These results suggested that HHS effectively inhibited LPS-induced NF-κB activation by blocking the nuclear translocation of NF-κB and the degradation of IκBα.

**Fig. 4:** Attenuation of LPS-induced NF-κB activation by HHS in RAW 264.7 macrophages. **a** The cells were treated with the indicated concentrations of HHS for 1 h before LPS treatment (100 ng/ml) for 30 min. Nuclear and cytosolic proteins were resolved on 10 % SDS-polyacrylamide gels, followed by Western blotting using anti-NF-κB p65 and anti-IκBα antibodies. Lamin B and actin were used as internal controls for the nuclear and cytosolic fractions, respectively. **b** Cells were pretreated with 300 μg/ml of HHS for 1 h prior to stimulation with LPS (100 ng/ml) for 30 min. Localization of NF-κB p65 was visualized with a fluorescence microscope after immunofluorescence staining with anti-NF-κB p65 antibody and an FITC-labeled anti-rabbit IgG antibody (green). Nuclei of the corresponding cells were visualized with DAPI (blue). **c** Following treatment with 300 μg/ml of HHS for 1 h, the cells were treated with 100 ng/ml of LPS for 30 min. Nuclear extracts were prepared, and the DNA binding activity of NF-κB was analyzed by an EMSA

### HHS attenuated LPS-induced AP-1 activation in RAW 264.7 macrophages

Inflammatory mediators and cytokines were mediated not only by NF-κB but also by another transcription factor, AP-1, which is activated by JNK [6, 7]. Several AP-1 family or CRE binding proteins have been shown to translocate to the nucleus during LPS stimulation [7, 12]. To evaluate the effect of HHS on the transcriptional activity of AP-1, the DNA-binding activity of AP-1 was measured by an EMSA. As depicted in Fig. 5a, treatment with LPS for 60 min increased the DNA-binding activity of AP-1 to its consensus DNA sequence. However, pretreatment with HHS attenuated this LPS-induced AP-1-DNA binding, suggesting that HHS inhibited AP-1 activity. Following inflammatory stimulation, the AP-1 heterodimers c-Jun and c-Fos are translocated into the nucleus, leading to the transcriptional activation of several inflammatory genes [7, 8]. We confirmed the inhibitory pattern of AP-1 by measuring the nuclear levels of c-Jun and c-Fos, in addition to their phosphorylation levels. As shown in Fig. 5b, when the cells were stimulated with LPS, the accumulation and phosphorylation of c-Jun and c-Fos markedly increased. However, upon HHS pretreatment, LPS-induced expression and phosphorylation of c-Jun and c-Fos was significantly attenuated (Fig. 5b). These results indicated that the anti-inflammatory effect of HHS on LPS-activated RAW 264.7 cells might occur through NF-κB, as well as AP-1, signaling pathways.

**Fig. 5:** Suppression of LPS-induced AP-1 activation by HHS in RAW 264.7 macrophages. **a** The cells were treated with 300 μg/ml of HHS for 1 h before LPS treatment (100 ng/ml) for 30 min. Nuclear proteins were resolved on 10 % SDS-polyacrylamide gels, followed by Western blotting using the indicated antibodies. Lamin B was used as an internal control for the nuclear fractions. **b** In a parallel experiment, nuclear extracts were prepared, and the DNA binding activity of AP-1 was analyzed by an EMSA

### Effects of HHS on the cell viability of LPS-stimulated RAW 264.7 macrophages

The effects of HHS on the viability of the RAW 264.7 cells were finally determined after incubation with or without LPS in the absence or presence of HHS. The relative cell viability was calculated by the absorbance of the untreated control group compared with the absorbance of each sample-treated group. The concentrations (100 to 300 μg/ml) of HHS used in this study did not show any cytotoxicity (Fig. 6), confirming that the anti-inflammatory potential of HHS in the LPS-stimulated RAW 264.7 cells was not due to any cytotoxic action of HHS.

**Fig. 6:** Effects of HHS and LPS on the cell viability of RAW 264.7 macrophages. The cells were treated with the indicated concentrations of HHS alone or pretreated with HHS for 1 h before 100 ng/ml of LPS treatment. After 24 h, the cell viability was assessed using an MTT reduction assay. Data are expressed as the mean ± SD of three independent experiments

### HHS suppressed LPS-induced phosphorylation of ERK and JNK in RAW 264.7 macrophages

MAPK signaling activated by phosphorylation plays an important role in NF-κB activation, and the inhibition of the MAPK pathway is sufficient to block the induction of proinflammatory factors by LPS [13, 25]. Thus, we examined the inhibitory effect of HHS on the activation of the MAPK pathway. To investigate whether HHS attenuated inflammatory responses through MAPK pathways, we assessed the effect of HHS on the LPS-induced phosphorylation of several MAPKs, including ERK, JNK, and p38 MAPK in RAW 264.7 cells. As shown in Fig. 7, ERK and JNK phosphorylation increased after the treatment with LPS for 30 min. However, pretreatment with HHS significantly attenuated the phosphorylation levels of these kinases compared with those of the LPS only-treated group. On the other hand, when the RAW 264.7 cells were stimulated with HHS alone, the level of phosphorylated p38 MAPK significantly increased, as it did with the LPS-only treatment. Moreover, HHS did not appear to have any effect on the LPS-induced phosphorylation of p38 MAPK. In addition, HHS did not affect the total forms of the three MAPKs, either in the presence or absence of LPS. These results indicated that the anti-inflammatory effect of HHS was possibly mediated via the blockage of ERK and JNK phosphorylation but that it was independent of the activation of p38 MAPK.

**Fig. 7:** Effect of HHS on LPS-induced phosphorylation of MAPKs in RAW 264.7 macrophages. The cells were pretreated with various concentrations of HHS for 1 h prior to exposure to LPS (100 ng/ml) for 30 min, and total proteins were isolated. The proteins were subjected to SDS-polyacrylamide gels, followed by Western blot analysis using the indicated antibodies and an ECL detection system

## Discussion

In this study, we evaluated the anti-inflammatory activities of HHS, a Korean traditional herbal formula, in LPS-stimulated RAW 264.7 murine macrophages in an attempt to source an anti-inflammatory agent from traditional medicinal resources with more effectiveness than current agents. Our results indicated that i) HHS significantly inhibited LPS-induced production of NO through the downregulation of iNOS expression; ii) HHS markedly suppressed LPS-induced release and expression of IL-1β and TNF-α; iii) HHS inhibited LPS-induced phosphorylation of ERK and JNK, but not p38 MAPK; iv) HHS attenuated the activation of NF-κB by blocking the nuclear translocation NF-κB and degradation of IkB; and v) HHS markedly inhibited LSP-induced activation AP-1 by suppressing the phosphorylation of c-Jun and c-Fos. The results presented in this study demonstrate that the underlying anti-inflammatory mechanisms of HHS are due, at least in part, to inhibition of LPS-induced activation of NF-κB, MAPK, and AP-1 signaling pathways.

The overproduction of proinflammatory mediators and cytokines by activated macrophages causes various inflammatory diseases [3, 26]. Therefore, identifying new agents capable of lowering the production of proinflammatory agents is regarded as an essential requirement for the alleviation of a number of inflammation-related disorders attributed to macrophage activation [12, 27]. In the present study, the production of NO was markedly elevated in response to LPS. However, the application of HHS inhibited the production of NO by LPS in a concentration-dependent manner (Fig. 1a). The results from the RT-PCR and Western blot analysis showed that pretreatment with HHS concentration-dependently reduced iNOS mRNA levels, with correlated reductions in the corresponding protein level (Figs. 1b and c). In addition, HHS was highly effective at inhibiting IL-1β and TNF-α production, which was associated with a reduction of mRNA and protein expression of IL-1β and TNF-α in the LPS-treated RAW 264.7 cells (Figs. 2 and 3). The present data indicated that HHS reduced mRNA levels of iNOS, IL-1β and TNF-α, which led to decreased protein levels of iNOS, IL-1β and TNF-α, and consequently reduced the quantities of NO, IL-1β and TNF-α that were produced by these enzymes.

The accumulated data demonstrates that specific transcription factors are mainly responsible for the transcriptional regulation of a variety of proinflammatory mediators and cytokines from activated macrophages [7, 10]. Among these, the NF-κB transcription factor family is a critical mediator of inflammatory processes. Thus, the inactivation of NF-κB in the immune system is a major therapeutic target for the downregulation of inflammatory responses. Along with NF-kB activation, AP-1 is able to regulate the expression of a large number of proinflammatory genes, which attract or activate immune cells [8, 11]. NF-κB and AP-1 is composed mainly of two proteins: p65 and p50 or c-Jun and c-Fos, respectively. In unstimulated cells, they exist in the cytosol in a quiescent form. Upon stimulation with LPS, they are activated and translocate to the nucleus where they activate their target genes by binding to their consensus sequences in their promoter regions. In addition to the NF-κB and AP-1 signaling pathways, MAPKs are a major group of signaling molecules that appear to play key roles in inflammatory processes because the phosphorylation of MAPK can stimulate the activation of NF-κB and AP-1 [27, 28]. Therefore, the MAPK signaling cascade is also an attractive therapeutic target for the development of treatments for inflammatory disorders.

In this study, Western blotting revealed that HHS was able to inhibit the LPS-evoked degradation of IkB and the nuclear translocation of NF-κB p65 (Fig. 4). Based on these results, we tested whether HHS inhibited NF-κB activity in RAW 264.7 macrophages by using an EMSA and found that HHS inhibited LPS-induced DNA-binding of NF-κB. To investigate whether the inhibition of NF-κB activation by HHS was associated with the MAPK pathway, the LPS-induced phosphorylation of various MAPKs family proteins, particularly ERK, JNK, and p38 MAPK, was assessed. The immunoblotting results revealed that HHS strikingly induced p38 MAPK phosphorylation, but it had no effect on the activity of ERK and JNK. In addition, the HHS pretreatment abolished the LPS-induced phosphorylation of ERK and JNK (Fig. 6). However, HHS failed to inhibit LPS-induced p38 MAPK phosphorylation, indicating that the anti-inflammatory responses by HHS may be independent on the p38 MAPK signaling pathway. In subsequent studies, the results from Western blotting of nuclear extracts indicated that HHS inhibited the expression and phosphorylation of c-Jun and c-Fos in LPS-challenged RAW 264.7 cells. Furthermore, the EMSA results demonstrated that the DNA-binding activity of AP-1 was significantly reduced in nuclear extracts obtained from LPS-activated RAW 264.7 cells that had been pretreated with HHS (Fig. 5). These results suggested that HHS blocked the binding of NF-κB and AP-1 to specific sequences of DNA, thereby preventing the formation of DNA/NF-κB and DNA/AP-1 complexes. In addition, changes in the phosphorylation of ERK and JNK might mediate HHS-induced inhibition of NF-κB and AP-1 transcriptional activities. In particular, deficiencies in the phosphorylation of these kinases could lead to decreases in the expression levels of inflammation-related genes.

## Conclusions

In conclusion, our findings showed that HHS effectively inhibited the LPS-induced production of proinflammatory factors, such as NO, IL-1β and TNF-α, in RAW 264.7 macrophages without causing cytotoxicity. A possible mechanism for this effect involves the ability of HHS to activate a signaling cascade, which results in the repression of NF-κB, ERK, and JNK and the activation of AP-1 in LPS-challenged macrophages. Although further investigation is needed to clarify the precise mechanisms by which HHS inhibits NF-κB and AP-1 activation and to identify the biologically active compounds of HHS responsible for the observed effects, HHS may be considered a potential therapeutic agent for the treatment of inflammation-related disease.
